The article "Molecular Docking and Green Synthesis of Bioinorganic TiO2 Nanoparticles against E.coli and S.aureus" was retracted in 2024. Reasons: signs of a paper mill; suspected computer-generated content; unreliable results or conclusions; concerns about the data.

# Molecular Docking and Green Synthesis of Bioinorganic TiO_2_ Nanoparticles against *E.coli* and *S.aureus*

**DOI:** 10.1155/2022/1142727

**Published:** 2022-10-15

**Authors:** Rasha Hamed Al-Serwi, Mohamed El-Sherbiny, T. V. Ajay Kumar, Abdulmalik Abdulghani Qasim, Thekra Khattar, Yahia Alghazwani, Ali Alqahtani, Venkatesan Krishnaraju, Jamal Moideen Muthu Mohamed, Venkatesa Prabhu Sundramurthy

**Affiliations:** ^1^Department of Basic Dental Sciences, College of Dentistry, Princess Nourah Bint Abdulrahman University, P.O. Box 84428, Riyadh 11671, Saudi Arabia; ^2^Department of Basic Medical Sciences, College of Medicine, AlMaarefa University, P.O. Box 71666, Riyadh 11597, Saudi Arabia; ^3^Azidus Laboratories Ltd., Rathinamangalam, Chennai 600048, Tamil Nadu, India; ^4^Department of Pharmacology, College of Pharmacy, King Khalid University, Guraiger, Abha 62529, Saudi Arabia; ^5^Vaasudhara College of Pharmacy, Sante Circle, Chintamani Road, Hoskote 562114, Karnataka, India; ^6^Centre of Excellence for Bioprocess and Bio Technology, Department of Chemical Engineering, Addis Ababa Science and Technology University, Addis Ababa, Ethiopia

## Abstract

This study used a simple solution evaporation approach to make a bioinorganic titanium dioxide (Bi-TiO_2_) photocatalyst for dye contaminant degradation. A variety of techniques, including *X*-ray diffraction (XRD), Fourier-transform infrared (FT-IR) spectroscopy, scanning electron microscopy (SEM) coupled with energy dispersive *X*-ray analysis (EDAX), and differential reflectance spectroscopy, had been employed to classify the structural and optical properties of the prepared bioinorganic photocatalyst (UV-DRS). Using simulated solar irradiation, the photocatalytic activity of the produced Bi-TiO_2_ nanoparticles was examined by detecting the degradation of a solution of methylene blue (MB) as a model dye molecule. The developed Bi-TiO_2_ photocatalyst demonstrates superior photocatalytic action than commercially available powder TiO_2_, according to photo-degradation experiments. E.*coli* and S.*aureus* bacterial strains were employed to assess the antibacterial activity of Bi-TiO_2_ nanoparticles. The most active molecules that gain antibacterial activity were examined in isolated or extracted components from the tulsi plant. The chosen compounds were docked with thymidylate kinase (TMPK), a potential therapeutic goal for the preparation of novel antibacterial drugs with the PDB ID of 4QGG. Five compounds, namely rosmarinic acid, vicenin-2, orientin, vitexin, and isoorientin, out of the 27 chosen compounds, showed a higher docking score and may aid in boosting antibacterial activity. The synthesized Bi-TiO_2_ nanoparticles produced antibacterial activity that was effective against Gram-positive bacteria. The nanomaterials that have been synthesized have a lot of potential in wastewater treatment and biomedical management technologies.

## 1. Introduction

Dyes are a type of coloring substance that is widely utilized in the textile industry, medicine, food, and cosmetics, among other things. When it comes to industrial applications, these dyes are discharged directly into the aquatic environment, posing a hazard to human life [1]. Dyes are classified into three groups: (i) cationic, (ii) anionic, and (iii) nonionic. Cationic dyes are utilized in a variety of industrial applications, including food coloring, pharmaceuticals, and textiles. When these cationic dyes are discharged directly into the aquatic system, they kill aquatic life by obscuring sunlight and reducing photosynthesis in the water. When humans drink dye-contaminated water, it causes vomiting, carcinogenesis, renal failure, and eye discomfort, among other things [2].

The dye material is removed using a variety of ways, including flocculation, adsorption, catalytic removal, filtering, and so on. Photocatalytic dye removal is one among them, thanks to its ease of synthesis, low cost, and high-efficiency materials are extensively utilized. Nanotechnology has developed a lot of consideration for the reason that, extensive kinds of uses in almost every sector, from textiles to medicine, and even electronics [3]. Nanomaterials are materials that have a nanoscale size in at least one dimension and substantial changes in properties and may be employed in a range of applications. Nanoscience and nanotechnology have been widely applied in the IT sector, energy, environment, aeronautics, medical, nanoscience, and biotechnology.

Several chemical processes are employed to generate smaller-sized metal oxide nanoparticles, including hydrothermal, sol-gel, coprecipitation, and solvothermal procedures. The toxicity of these chemically generated bioinorganic titanium dioxide (Bi-TiO_2_) nanoparticles is a key stumbling hurdle when employing them for biological purposes. To employ Bi-TiO_2_ nanoparticles in biological applications, biological processes are exploited to manufacture Bi-TiO_2_nanoparticles that are less or nontoxic. Algae biosynthesize Bi-TiO_2_ nanoparticles [4], but the time-consuming procedure and limited availability of microorganisms limit their use in biological applications.

Herbal extracts containing phytochemicals, particularly from leaves, are frequently used to produce Bi-TiO Bi-TiO_2_2 nanoparticles because of their abundant availability, quick synthesis, and potential to make smaller stable nanoparticles [5]. Bi-TiO_2_nanoparticles have been used in several products, including skin care treatments, food coloring, inks, and toothpaste. These Bi-TiO_2_ nanoparticles may be the application on the photocatalytic material for the breakdown of numerous organic compounds to a greater degree by reducing the band gap. Bi-TiO_2_ creates higher dynamic types for organic molecule breakdown when exposed to UV/visible light. Because of its simple and ecologically benign synthesis procedure, the photogenic production of Bi-TiO_2_ nanoparticles has sparked a lot of attention [6].

*Ocimum sanctum* (tulsi) is medicinal basil widely used throughout Asia, Africa, and the Arab world. The leaves of *Ocimum sanctum* have long been used to cure a range of infections. *Ocimum sanctum* is a member of the Lamiaceae family, and its leaves contain several chemical compounds such as ursolic acid, eugenol, oleanolic acid, rosmarinic acid, linalool, carvacrol, and -caryophyllene. The presence of phenolic eugenol matrix is responsible for the decrease of Ca and Co metal ions by leaf extract. According to Apsana et al., SrO-NPs generated utilizing a microwave green chemical technique have superior antibacterial activity [7].

Molecular docking is a well-organized approach that aids in the calculation of the ligand's leading binding modes and the structure of a three-dimensional protein. The ability to anticipate binding modes is critical for revealing significant structural properties and interactions, as well as providing helpful data in the development of effective inhibitors [8]. A ligand is a tiny molecule that may engage with a protein's binding sites in one of several potential conformations. Binding modalities are the methods through which binding takes place. Molecular docking is commonly used in contemporary drug design to detect drug data and concern receptor interactions. It is often employed to determine the binding affinity, orientation, and activity of drug nominees concerning a target protein [9]. The current study builds on previously reported components extracted from tulsi (*Ocimum sanctum Linn*) extract to assess its antibacterial efficacy and serve as a foundation for future research. The leaf extract of *Ocimum sanctum* was employed to make Bi-TiO_2_ nanoparticles in this study. FTIR, SEM, EDAX, and XRD analyses are used to characterize the nanoparticles. S.*aureus*, *E. coli*, and MB dye were used to test the bacterial and catalytic strength of Bi-TiO_2_ nanoparticles.

In the proposed work, the facile and economical production of Bi-TiO_2_ nanoparticles was achieved through green synthesis. In the current study, titanium tetra isopropoxide and *Ocimum sanctum* leaf extract were combined to create Bi-TiO_2_ nanoparticles using a solvothermal method. After SEM examination, it was discovered that the Bi-TiO_2_ nanoparticles had a spherical shape and an aggregated appearance. FTIR results show that Bi-TiO_2_ nanoparticles are pure. The produced Bi-TiO_2_ nanoparticles were found to have more photocatalytic degradation capacity than the MB dye. In addition, Bi-TiO_2_ nanoparticles have strong antibacterial action against Gram-positive bacteria and showed potential as a candidate for methylene blue degradation under simulated sun irradiation.

## 2. Materials and Methods

### 2.1. Plant and Chemicals

The plant compounds (*Ocimum sanctum* leaf) were obtained from the Tiruchirappalli local market in Tamilnadu, India. Double distilled water was used to treat the raw material of titanium (IV) isopropoxide (Merck 99% purity). Methylene blue (MB) solution was obtained from Loba Chemicals in Mumbai, India. The rest of the chemicals and reagents were of high-grade analytical quality.

### 2.2. Molecular Docking

To assist our research, phytochemical or bioactive ingredients extracted from tulsi (*Ocimum sanctum Linn*) were chosen at random.  Table 1 shows a list of 27 phytochemical compounds that have been identified in the literature [10,11], and they were tested for antibacterial activity using molecular docking research.  Figure 1 shows the structures of the compounds that were chosen. The Schrodinger suite program was used to dock 27 chemicals against the protein thymidylate kinase (TMPK) from *Staphylococcus aureus*.

#### 2.2.1. Preparation of Ligand

The LigPrep module's scripts offer effective methods for creating ligands both continuously and in batches [12]. It can also make amazing 3D structures from a variety of chemicals that resemble drugs. In addition, it creates unique, low-energy 3D structures for every key with precise chiralities. It examines the stereochemistries, tautomers, ring conformations, and ionization states of the ligands. In addition, it filters out molecules according to several criteria, such as molecular weight, particular quantities, and the presence of functional groups. ChemOffice was used to create a drawing of tulsi that contained 27 different compounds. The SDF file was then saved and imported into Schrodinger's LigPrep module. [13]. ChemOffice is a scientifically intelligent, integrated suite of personal productivity tools that assists scientists in effectively managing their workload, comprehending their data more thoroughly, and producing scientific reports in an expert and timely manner.

#### 2.2.2. Preparation of Proteins and Construction of Receptor Grids

The three-dimensional (3D) crystal structures of *Staphylococcus aureus* thymidylate kinase (TMPK) were found in the Protein Data Bank database (PDB : ID 4QGG) [14]. For exact energy measurement, Glide uses a script called “all-atom force field.” Glide additionally reorganizes the missing side chains with steric conflicts, aligning and allocating suitable bond ordering and ionization states. The Protein Preparation Wizard module of the Schrodinger suite was utilized to complete the procedure in its entirety.

The respective pair of receptor fields was represented as a grid with a form and characteristic that consistently allows for more precise ligand pose scoring [15]. The options in every tab of the receptor network group panel aid in describing the receptor's structure by omitting a few cocrystallized ligands if they are available. Similarly, it helps to set up Glide restrictions by identifying the active site's location and figure as “receptor grids” [16].

#### 2.2.3. Ligand Docking

A single or many ligand structures, as well as previously established receptor glides, are required for the ligand docking process. Glide employed an E-model scoring method to find the optimal protein-ligand complexes for a ligand and a Glide score function to order the compounds to distinguish between ligands that have strong bonding (actives) and those that have weaker bonding (inactive) with proteins [17]. It is known as the lowest-scoring chemical and is thought to be the most effective against the protein. For the ligand docking investigation, Schrödinger Suite's Glide XP (extra precision) module was employed. The ligand's glide or docking score aids in the classification of molecules based on their capacity to interact.

### 2.3. Preparation of *Ocimum sanctum* Leaf Extract

For 24 hours, fresh *Ocimum sanctum* leaves were repeatedly rinsed with demineralized water at room temperature. 500 mg *Ocimum sanctum* leaves were added to 200 mL distilled water in a 500 mL beaker and cooked for one hour at 100°C, and filtered leaf aliquots were collected for further research.

### 2.4. Synthesis of Bioinorganic Titanium Dioxide Nanoparticles (Bi-TiO_2_ NPs)

1 M titanium tetra isopropoxide was added to a 250 mL beaker containing 20 mL *Ocimum sanctum* leaf extract, which was agitated for 4 hours at 60°C. After that, the entire solution was centrifuged for 600 seconds at 12000 rpm after the reaction. The Bi-TiO_2_nanoparticles were then rinsed repeatedly with ethanol and centrifuged for 300 seconds at 8000 rpm. Finally, the separated Bi-TiO2nanoparticles were calcined in a furnace at 500°C for around 3 hours, using a 5°C/min ramp [18]. Further analytical procedures were performed using the sintered titanium dioxide nanopowder. Titanium dioxide is both absorbent and odorless. In powder form, its primary application is as a common pigment that adds whiteness and opacity. Porcelain enamels have been given brightness, hardness, and acid resistance thanks to the employment of titanium dioxide as a bleaching and opacifying agent. As starting materials, titanium tetraisopropoxide, isopropanol, and deionized water were employed. After calcination at 400°C, TiO_2_ nanopowder was produced by carefully controlling the relative amount of the precursor materials, the pH, and the peptization duration. To study the impacts of sintering on nanopowder particles, densification behavior, phase evolution, and mechanical properties, as-synthesised powder was uniaxially compacted and sintered at an increased temperature of 1100–1600°C.

### 2.5. Characterization of Bi-TiO_2_Photocatalyst

The patterns of *X*-ray diffraction (XRD) were checked to utilize (PANalytical B. V., Netherlands). A powder sample approach was used to examine the composite Fourier-transform infrared (FT-IR) spectra, which ranged from 400 to 4000 cm-1 [19–21]. Scanning electron microscopy (SEM) combined with EDAX with a 30 kV accelerating voltage was applied to evaluate the surface morphology of the composite samples (Carl Zeiss). Using BaSO4 as a reference, UV-vis diffused reflectance spectra were scanned using a spectrophotometer (UV-2700, Shimadzu, Japan).

### 2.6. Photocatalytic Dye Degradation Activity

Using simulated solar irradiation, the photocatalytic degradation of MB dye was used as a photocatalyst for Bi-TiO_2_. Due to its particular benefits over traditional water treatment methods, photocatalysis is one of the sophisticated oxidation technologies that are attracting more and more attention. TiO_2_ semiconductor photocatalysis has demonstrated tremendous promise for the removal of a variety of chemical and microbiological contaminants. Only the UV area is where TiO2 absorbs (band gap: 3.2 eV). A green process requires the least amount of energy possible, making solar light the main source of photo energy. While the majority of solar insolation is in the visible wavelengths, only around 5% of the total energy in solar radiation is in the UV area. By narrowing its band gap, a catalyst can be made to absorb visible light. As a result, visible light photocatalysis has drawn the attention of the scientific community. Doping TiO_2_ has improved its ability to absorb visible light. In prior reports, several transition metal ions were looked into as dopants. It has been found that varied dopant positions in the host matrix control the photocatalytic capabilities of TiO2. To begin the reaction, a 250 mL beaker was filled with 50 mL of MB dye solution (1x10-5 M). The distance between the simulating light and the dye solution is around ten centimeters [22]. To attain the adsorption-desorption equilibrium, 0.05 gm of the photocatalyst was added to the dye solution and kept dark for 2 hours. After reaching equilibrium, the solution was stirred continuously at 550 rpm for 30 minutes before being put in a simulated sun simulator. The aliquot solution was then collected every 10 minutes, centrifuged, and the dye degradation was determined using a spectrophotometer and the absorbance value of MB. The removal % of the dye molecule was determined using the following calculation:

(1) $$\begin{array}{c} \text{Percentage of dye }de\;g\text{ radation}=\left(CMBi-\frac{CMBT}{CMBi}\right)x\text{,} \end{array}$$

where C_MBi_ = initial dye concentrations. **C**_MB**T**_ = concentration of dye solution at time interval ‘t'.

### 2.7. Antibacterial Activity

The antibacterial susceptibility of *Ocimum sanctum* leaf and Bi-TiO_2_ nanoparticles is assessed using the disc diffusion technique. The antibacterial capabilities of tulsi extract and Bi-TiO_2_ nanoparticles were investigated using Gram-positive and Gram-negative bacteria as model microorganisms, such as *E. coli* and *S. aureus* [23]. To prepare the nutritional agar plate, all glassware is sterilized in a 120°C autoclave for 30 minutes. Circular discs impregnated with 100 *µ*L of produced Bi-TiO_2_ nanoparticle and *Ocimum sanctum* leaf were put in the well of the Petri plates using a cork borer. The sample-inoculated dishes were incubated for 24 hours at 40°C. After the incubation time has ended and all plates have displayed the zone of inhibitions (ZOI), the ZOI was measured in mm scale using a ruler.

## 3. Results and Discussions

### 3.1. Molecular Docking Outcomes

Using in silico molecular docking experiments, the current bioactive components of tulsi (*Ocimum sanctum Linn*) were randomly selected to assess their antibacterial efficacy. About 27 compounds were chosen for the study based on it, and they were identified and obtained from the PubChem website in .SDF format. For the docking investigations, the compounds' two-dimensional (2D) structures were converted into three-dimensional (3D) constructions. The geometrical optimization was performed using the force field OPLS-2005 using condensed newton conjugate gradient (TNCG) reduction. Using the force field OPLS2005, the ligands are generated using LigPrep with Epik [24] by 7 2.0 pH units to supplement protonation and tautomeric positions. For each ligand, the stereoisomers of the low-energy complexes were predicted, and the one with the lowest-energy 3D structure was retained.

Moreover, the protein data library provided the 3D modeled structure (4QGG) of thymidylate kinase (TMPK) from *Staphylococcus aureus*. The protein was made with the Schrodinger suite's “protein preparation wizard” function. The centroid of active site residues was used to build a grid using the van der Waals scaling factor of 1.0 and the fractional charge cutoff of 0.25 after the protein was prepared.

Ligand docking was performed with the produced protein thymidylate kinase and the 27 ligands utilizing Schrodinger maestro's “Ligand docking.” Following successful docking, characteristics such as the docking score, ECoul (Coulomb energy), Glide evdw (Van der Waals energy), Glide energy, and interacting remains (hydrogen bond/- bond) were prioritized and discovered. The summit of collaboration among the ligands and the protein was measured using these characteristics.  Table 2 shows the expected relative scores for the docking score, Glide ECoul, Glide evdw, interacting residues, and Glide energy. The docking score or glide score with the lowest or least score or energy was supposed to be the maximum effective attraction in the direction of the protein [25].

Based on the data (Table 2), the majority of chemicals exhibit a high affinity for the protein thymidylate kinase. Rosmarinic acid, vicenin-2, orientin, vitexin, and isoorientin were found to have a higher affinity for the protein than the others. The docking scores of rosmarinic acid, vicenin-2, orientin, vitexin, and isoorientin are, respectively, −11.45, −11.02, −10.68, −10.27, and −8.69.

The amino acid residues ARG48, SER96, GLN101, and 4(HOH) have well-built hydrogen bond interactions with the chemical rosmarinic acid. Rosmarinic acid's Glide evdw, ECoul, and Glide energy were −25.73, −28.73, and −54.45, respectively. Vicenin-2 has a docking score of −11.02, and hydrogen bond interactions with amino acids such as SER96 and HOH have been detected. Vicenin-2 ECoul, Glide evdw, and Glide energy were −31.71, −21.47, and −53.18, respectively. Orientin, with a docking score of -10.68, had more hydrogen bond interactions with the amino acid residues GLN101 and HOH, and its ECoul, Glide evdw, and Glide energy were −28.82, −21.82, and −50.64, respectively.

Furthermore, the other chemicals had strong hydrogen bond interactions but had a lower protein binding affinity. As a result, the compounds are predicted to have higher binding affinity because their donor or acceptor on the side groups/chains creates hydrogen bonds with residues. All 27 substances were shown to have binding characteristics to the protein thymidylate kinase. To summarize these findings, rosmarinic acid > vicenin-2 > orientin > vitexin > isoorientin was the top-scoring chemical based on docking scores against the bacterial marker.

### 3.2. FTIR Analysis

The chemical skeleton of the biosynthesized Bi-TiO_2_ nanoparticles was studied using FTIR spectroscopy, and it has important functional groups.  Figure 2(a) shows the FTIR spectrum of the generated Bi-TiO_2_photocatalytic nanoparticle. The bands 3415 and 1631 cm^−1^ were indexed to the hydroxyl (O–H) group's asymmetric and symmetric stretching vibrations, respectively, and specified the presence of moisture in the sample. The typical peak of the O–Ti bond and Ti–O–Ti bond in the Bi-TiO_2_ matrix is 712 cm^−1^ [26]. The vibrational modes of O–H, RCOO^−^, and C–C groups present in the processed Bi-TiO_2_ sample match the weak bands about 2930 and 2852 cm^−1^, indicating that these groups were not completely removed after ethyl alcohol and demineralized water washing. C=O and–CH_2_- groups, which are present in the produced Bi-TiO_2_ nanoparticles, might also be responsible for the peaks at 1384 cm^−1^.

### 3.3. XRD Analysis

Figure 2(b) displays the XRD pattern of the synthesized Bi-TiO_2_ photocatalyst sample. Diffraction peaks (101), (004), (200), (105), (211), (204), (118), and (315) are assigned to appropriate crystal planes of powder Bi-TiO2 according to JCPDS card no. (21–1272). The diffraction peak found is clearly defined and points to the Bi-anatase TiO_2_s phase. These anatase phases are well-known in water purification and color removal processes [27]. The size of the Bi-TiO_2_ photocatalyst was determined using the Debye Scherrer formula and is 24 nm. The existence of a pure anatase phase in the XRD pattern indicates that there are no additional impurities connected to the rutile phase, suggesting sample purity.

### 3.4. UV-DRS Analysis

An essential factor in defining the photoactiveness of photocatalytic materials is their optical absorption properties. The bandgap energy spectra and absorption spectra of Bi-TiO2 are displayed in Figure 3(a). The excited charge carriers in the 2-p state were revealed by the Bi-TiO_2_ nanoparticles' absorption in the UV spectrum. The direct bandgap energy value for the produced Bi-TiO_2_ photocatalyst is determined using the suggested Tauc plot approach. The quantities hv (the photon energy) and (h)1/2 (stands as the material's absorption coefficient) are displayed on the ordinate and abscissa, respectively, of the Tauc plot. The energy of the optical bandgap of the amorphous material can then be obtained by extrapolating this linear region to the abscissa.  Figure 3(b) shows that the created composite had a smaller bandgap value than commercial Bi-TiO_2_ (3.15 eV) [28], indicating improved light absorption and greater conductivity. Bi-TiO_2_ photocatalyst can therefore be employed in visible light photocatalysis. Although TiO_2_ has a number of advantages over other semiconductor photocatalysts, its 3.2 eV band gap prevents it from being used in the UV area of the electromagnetic spectrum (387.5 nm). As a result, one of the main difficulties in the field of semiconductor photocatalysis is the development of visible light active titanium dioxide.

### 3.5. Morphology

Figures 4(a) and 4(b) show typical SEM images of Bi-TiO_2_ nanoparticles at higher (a) and lower (b) magnifications, respectively. In both lower and higher magnifications, spherical aggregated particle Bi-TiO_2_ with smooth surface forms bigger particles [29]. The average particle size of ordinary titanium dioxide is 0.20 m. In the current study, we see that a sizable region was covered in homogenous, sphere-like Bi-TiO_2_ nanoparticles with a particle size of roughly 100 nm. The big aggregative particles may be seen in the plant nutrients that are already present. The nanoparticles are aggregated and shuffled together due to the presence of plant chemicals.

### 3.6. EDX Analysis

FTIR analysis was used to examine the present plant nutrients and their stretched molecules.  Figure 4(c) shows the EDX spectrum of the studied Bi-TiO_2_ samples, which revealed peaks of Ti and O elements.  Figure 4(d) shows that the existence of Ti (43.12) and O (58.88) atomic weight percentages substantiates the synthesis of pure Bi-TiO_2_with no additional impurities, which was the reliable argument with the XRD and FTIR results.

### 3.7. Photocatalytic Activity

In chemistry, a scavenger is a chemical that is introduced to a mixture to eliminate or deactivate contaminants and undesired reaction products, such as oxygen, in order to prevent any negative reactions. It is important to have a hole scavenger present during photocatalytic reduction reactions, which is often an organic chemical. Since it competes with the substrate for photogenerated electrons, oxygen is often undesirable in the photoreduction process.

Under simulated sun irradiation for 120 minutes, the photocatalytic activity of Bi-TiO_2_ nanoparticles over cationic methylene blue dye was depicted in Figure 5(a), which illustrates the percentage of MB dye elimination under hazy and illumination circumstances utilizing photo catalyst Bi-TiO_2_. Adsorption followed by photocatalytic elimination of MB dye occurred as a result of the dual action of photocatalytic Bi-TiO_2_. Figure 5(a) shows that the photocatalytic removal % is high, while the adsorption percentage is low, which is owing to the Bi-TiO_2_ photocatalyst having fewer adsorption sites. By plotting the time of irradiation vs ln C/C0, the kinetic analysis reviles the discoloration of MB using the *k* app the first-order kinetics utilizing the straight line displayed in Figures 5(b) and 5(c). The apparent rate constant of dye molecules under the effect of simulated solar light irradiation is calculated using the following formula [30]:

(2) $$\begin{array}{c} \ln\frac{C0}{C}=\text{kapp}.t\text{,} \end{array}$$

Figure 5(d) shows the photocatalytic degradation efficiency during the first cycle, which was 94 percent (d). In alternate cycles 2, 3, 4, and 5, the catalyst activity reduces marginally, resulting in dye degradation efficiency of 92, 91, 90, and 88 %, respectively.

The kinetic rate constants for commercial Bi-TiO_2_ nanoparticles and synthesized Bi-TiO_2_ catalysts were chosen to be 0.0134 min1 and 0.02414 min1, respectively. The produced Bi-TiO_2_ surface has an anatase crystalline phase, which is a promising candidate for the destruction of different colored stains. The current study effort was compared to the previously published work, and the outcomes were listed in Table 3. The photolysis process starts when exposed to simulated solar radiation once the environment has reached a state of adsorption-desorption kinetic equilibrium. By replicating the oxidation reduction brought on by the surface contact with the Bi-TiO_2_ catalyst during the photocatalytic degradation phase of the MB molecules, it promotes the photo-produced hole and OH radicals to the MB molecules. It was customary to time the synthesis of CB (*e*) in the transmission band and VB h+ in the valence band to coincide with the simulated light energy that revealed the Bi-TiO_2_ surface. These generated electrons react with water molecules in a hurry to create a chain of highly reactive radical species (OH−) and (•O2−), which are responsible for the breakdown of a significant amount of MB molecules, as shown in Figure 6. The deactivation of the photocatalyst is caused by surface poisoning of the system by adsorbed intermediates [33].

(3) $$\begin{array}{c} {\text{TiO}}_{2}{+\text{hv}®\text{TiO}}_{2}{.\text{VB}}^{h+}+\text{Bi}-{\text{TiO}}_{2}C.B\left(e-\right)\text{,} \end{array}$$

(4) $$\begin{array}{c} {\text{TiO}}_{2}{V.B}^{\left(h+\right)}{+H}_{2}{O®\text{TiO}}_{2}{+H}^{+}+\text{OH}-\left(\text{Radicle}\right)\text{,} \end{array}$$

(5) $$\begin{array}{c} {\text{TiO}}_{2}C.B\left(e-\right){+\text{OH}}^{-}{®\text{TiO}}_{2}+.\text{OH,} \end{array}$$

(6) $$\begin{array}{c} \text{Ti}O_{2}^{h+}{+O}_{2}®O2\text{,} \end{array}$$

(7) $$\begin{array}{c} O_{2^{\cdot }}+\frac{\text{OH}}{h^{+}}{+C16H18\text{ClN}3S}^{.+}+⟶\text{Degradation }{\text{products}+H}_{2}{O+\text{CO}}_{2}\text{.} \end{array}$$

### 3.8. Antimicrobial Activity

Figure 7 shows the results of testing the produced Bi-TiO_2_ nanoparticles and *Ocimum sanctum* leaf extract with microbiological species such as *S. aureus* and *E. coli*. The antibacterial activity of the *Ocimum sanctum* leaf extract and manufactured Bi-TiO_2_ against *S. aureus* (3.6 mm) and *E. coli* (4.1 mm) was substantial (5.1 mm). The greatest inhibition zone was created by Bi-TiO_2_ nanoparticle over *E. coli* (7.9 mm) bacterium when the inhibition zone of plates was measured. A sum of three tests is carried out and the action of synthesized Bi-TiO_2_ generated hydroxyl groups and reactive oxygen species (ROS), which are capable of melting the cell wall because phospholipid peroxidation of bacteria leads to death [41, 42], is the mechanism of this well-developed antibacterial activity. In this paper, Bi-TiO2nanoparticles are shown to be an effective antimicrobial medicine that can pave the way for the development of novel antimicrobial pharmaceuticals and agents.

The application of organic carbon-based compounds as performance boosters in photocatalysis should be investigated in addition to inorganic doping components such as rare-earth metal/metal/nonmetal sources. This is a promising technique, according to the findings that have already been reported and evaluated in this work. Such C-based compounds are also presenting a different option for nonprecious metal dopants. But in order to effectively reduce CECs, this new strategy of C-based compound-enhanced photocatalytic materials needs in-depth research on the processes, destiny, and toxicity of end products that, in some situations, may even be more toxic than the parent molecule. There is a need for additional research in this area and as part of the mineralization investigations. It is important to correctly identify the deteriorated products and determine how well the utilized catalyst can break down both the parent component and the degraded end products. The addition of elements from outside the system further complicates the already complex heterogeneous photocatalysis process. The majority of research in such systems contains cocatalysts, tricatalysts, heterostructures, sacrificial agents, chemical scavengers, and so on; as a result, a stringent catalytic reaction mechanism is envisaged. There is a need to do more in-depth research in this area because the mechanism of composite semiconductor photocatalysts is still not fully understood, particularly with regard to the charge transport carriers, interactions, and underlying associated mechanisms occurring in these systems. There is a need to concentrate on understanding the economic aspects of the various systems with respect to the operational cost of running them either as a single AOPs system or as a combined system in the lead up to fully deployable and operational pilot plants for the removal of CEC compounds from actual wastewater, especially given the high level of AOPs studies that have already been performed, particularly in the area of water/wastewater decontamination. In addition, rather than being restricted to laboratory settings and systems, the use of synthetic photocatalyst materials should be tested against a wider range of wastewater matrix samples with a variety of untargeted pollutants. Research should refrain from employing the target compound surrogate that is created when the parent molecule is dissolved in synthetic samples manufactured with ultrapure water as the solvent. Although the use of dye compounds as solar spectrum sensitizers and energy scavengers by the photocatalytic materials that are connected well has gained considerable attention, however, specific information regarding the charge transport mechanism in these compounds is still unknown, necessitating further research for a clearer understanding. In order to improve these sensitizers' water solubility, thermal resilience, and ability to be used in a more environmentally friendly way, additional study must focus on the synthesis and purification of the best performing functional group of the macrocyclic rings [43–53].

## 4. Conclusion

In conclusion, green synthesis was employed to create Bi-TiO_2_ nanoparticles simply and cost-effectively. Using a solvothermal technique, Bi-TiO_2_nanoparticles were mixed from titanium tetra isopropoxide and *Ocimum sanctum* leaf extract in the current work. The Bi-TiO_2_ nanoparticles were found to have a spherical shape and an aggregated appearance after SEM inspection. The purity of Bi-TiO_2_ nanoparticles is confirmed by FTIR findings. The photocatalytic degradation potential of the synthesized Bi-TiO_2_ nanoparticles was found to be superior to that of the MB dye. Finally, Bi-TiO_2_ nanoparticles showed promise as a candidate for methylene blue degradation under simulated solar irradiation and have excellent antibacterial activity against Gram-positive bacteria. As a result, the selected tulsi structures were evaluated for their binding approach against the protein thymidylate kinase (TMPK) from *Staphylococcus aureus*, which has been proven to have shown a key role in bacterial resistance. The best-docked substances for the marker thymidylate kinase were rosmarinic acid, vicenin-2, orientin, vitexin, and isoorientin (TMPK). These chemicals might be used to create novel gifted molecules that help inhibit the *Staphylococcus aureus* protein thymidylate kinase (TMPK). The current findings suggest that Bi-TiO_2_ nanoparticles are an efficient photocatalytic agent for pollution cleanup in various dye-based industries.

## Figures and Tables

**Figure 1:** (a) The identified bioactive compounds and the chemical structures in tulsi (*Ocimum sanctum Linn*). (b): The identified bioactive compounds and the chemical structures in Tulsi (*Ocimum sanctum Linn*).

**Figure 2:** (a) FTIR spectrum and (b) XRD pattern of synthesized Bi-TiO_2_nanoparticle.

**Figure 3:** (a) UV-DRS and (b) bandgap spectrum of synthesized Bi-TiO_2_nanoparticle.

**Figure 4:** (a and b) SEM images, (c) EDX spectrum, and (d) the table of synthesized Bi-TiO_2_nanoparticle.

**Figure 5:** (a) Photocatalytic MB dye degradation efficiency, (b) C/C0, (c) ln C/C0 vs time, and the (d) reusability study of Bi-TiO_2_ nanoparticle.

**Figure 6:** Schematic representation of MB dye degradation mechanism.

**Figure 7:** Antibacterial activity of Bi-TiO_2_ nanoparticles and *Ocimum sanctum* leaf extract over Gram-positive and Gram-negative bacteria.

**Table 1:** The identified phytochemical compounds in the literature.

S. No	Name of the compound	S. No	Name of the compound
1	4,5-Dihydroxy-7,8-dimethoxyflavone	15	Isoorientin
2	Apigenin	16	Isovitexin
3	Beta-caryophyllene	17	Linalool
4	Beta-elemene	18	Luteolin
5	Beta-sitosterol	19	Molludistin
6	Bieugenol	20	Myrtenal
7	Carnosic acid	21	Oleanolic acid
8	Carvacrol	22	Orientin
9	Cirsilineol	23	Rosmarinic acid
10	Cirsimartin	24	Stigmasterol
11	Citrusin C	25	Ursolic acid
12	Dehydrodieugenol	26	Vicenin-2
13	Eugenol	27	Vitexin
14	Germacrene D		

**Table 2:** The docking score, ECoul (Coulomb energy), Glide evdw (van der Waals energy), interacting residues, and the type of interaction of 27 bioactive substances with the protein thymidylate kinase were calculated (TMPK). The docking scores were determined using Schrodinger Maestro Glide software (version 2018.1), where HB stands for hydrogen bonding and Pi-Pi stands for a -bond.

Target protein	Name of the compound	Docking score	Glide ECoul (coulomb	Glide evdw (kcal/mol	Glide energy (coulomb	Interacting residues (HB/Pi-Pi)
4QGG	4,5-Dihydroxy-7,8-dimethoxyflavone	−4.54	−5.05	−27.85	−32.90	ARG70/PHE66 and TYR100
	Apigenin	−4.50	−9.08	−22.54	−31.62	ARG48/3(HOH)
	Beta-caryophyllene	−2.15	−1.11	−11.78	−12.89	—
	Beta-elemene	−2.56	0.14	−13.99	−13.86	—
	Beta-sitosterol	−3.79	−7.16	−22.67	−29.83	THR16
	Bieugenol	−**5.66**	−5.99	−21.32	−27.31	GLU37, ARG48 and HOH
	Carnosic acid	−4.44	−9.94	−8.65	−18.59	GLU37, ARG48 and 2(HOH)
	Carvacrol	−4.31	−3.14	−19.39	−22.53	ARG70 and SER97
	Cirsilineol	−4.96	−6.53	−29.93	−36.47	ARG92 and ARG97/PHE66 and TYR100
	Cirsimartin	−4.56	−6.97	−25.67	−32.64	SER97/TYR100
	Citrusin C	−**7.90**	−16.83	−12.97	−29.80	ARG36, ARG48 and HOH
	Dehydrodieugenol	−**6.14**	−12.16	−21.86	−34.02	ARG36 and ARG48 and 2(HOH)
	Eugenol	−4.86	−5.62	−21.37	−26.99	SER97/TYR100
	Germacrene D	−3.04	−0.18	−13.14	−13.32	-
	Isoorientin	−**8.70**	−17.56	−25.95	−43.51	2(HOH)
	Isovitexin	−**7.31**	−18.99	−25.42	−44.41	TYR100 and HOH
	Linalool	−2.85	−6.17	−13.69	−19.86	ARG48 and HOH
	Luteolin	−**5.14**	−7.41	−26.85	−34.26	PHE66 and ARG70/PHE66 and TYR100
	Molludistin	−**8.12**	−13.68	−28.34	−42.02	ARG48 and HOH
	Myrtenal	−4.34	−6.45	−16.27	−22.71	ARG70 and SER97
	Oleanolic acid	−**5.10**	−18.56	−13.29	−31.86	GLY12, ARG36, ARG48 and 2(HOH)
	Orientin	−**10.68**	−21.82	−28.82	−50.64	GLN101 and 2(HOH)
	Rosmarinic acid	−**11.45**	−28.73	−25.73	−54.45	ARG48, SER96, GLN101 and 4(HOH)/PHE66
	Stigmasterol	−3.27	−5.21	−17.72	−22.93	-
	Ursolic acid	−4.38	−17.56	−10.81	−28.37	ARG36 and ARG48 and 3(HOH)
	Vicenin-2	−**11.02**	−21.47	−31.71	−53.18	SER96 and HOH
	Vitexin	−**10.27**	−24.46	−22.84	−47.29	GLN101 and 3(HOH)

**Table 3:** Comparison with collected work results.

S.No	Catalyst	Pollutant	Dye/Catalyst dosage	Irradiation source	Efficiency (%)	Ref
1.	RGO/TiO_2_	Diphenhydramine (DP) and methyl orange	7.5 mL/1.0 g L−1	Mercury	94	[31]
2.	Sn/TiO_2_	Malachite green	25 ml	UV	90	[32]
3.	Pd/TiO_2_	Methylene blue	0.75 g/500 ml	Xenon 300 W	99.5	[33]
4.	CeO_2_/TiO_2_	Bromophenol dye		Xenon 300W	72	[34]
5.	TiO_2_nanotubes	Indigo carmine	100 ml/0.1 g/L	Mercury 125W	90	[35]
6.	TiO_2_/C	Blue QR 19	200/50 mg	Mercury 125 W	89	[36]
7.	Ag-coated ni@ TiO_2_	Crystal violet	20 mL/10 mg	Hg lamp20 W	80	[37]
8.	TiO_2_	Methyl orange	50 mL	Xenonlamp150 W	80	[38]
9.	RuO_2_/SiO_2_/TiO_2_	Methyl orange	4 ml	F15 W/T8 UV	98	[39]
10.	CNT/TiO_2_	Methyl orange	1000 mL/200 mg	Mercury300 W	94	[40]
11.	Bi–TiO_2_	Methylene blue	50 ml/0.05 mg	Xenon arc lamp	95	Current work

## Data Availability

The datasets used and/or analyzed during the current study are available from the corresponding author upon reasonable request.
